The article "Genetic variation and diversity in 199 Melilotus accessions based on a combination of 5 DNA sequences" was retracted in 2020. Reasons: errors in the data; duplicated data; duplicate publication.

# Genetic variation and diversity in 199 *Melilotus* accessions based on a combination of 5 DNA sequences

**DOI:** 10.1371/journal.pone.0194172

**Published:** 2018-03-13

**Authors:** Hongxiang Zhang, Fan Wu, Wenli Guo, Rong Bai, Zhuanzhuan Yan, Blaise Pascal Muvunyi, Qi Yan, Yufei Zhang, Xianfeng Yi, Jiyu Zhang

**Affiliations:** 1 State Key Laboratory of Grassland Agro-ecosystems; Key Laboratory of Grassland Livestock Industry Innovation, Ministry of Agriculture; College of Pastoral Agriculture Science and Technology, Lanzhou University; Lanzhou, China; 2 Guangxi Institute of Animal Sciences, Nanning, China; National Cheng Kung University, TAIWAN

## Abstract

*Melilotus* is an important genus of legume plants and an herbage with excellent nitrogen fixation; it can tolerate extreme environmental conditions and possesses important medicinal value. However, there is limited genetic information about the genus; thus, we analysed four chloroplast loci (*rbc*L, *mat*K, *psb*A-*trn*H and *trn*L-F) and one nuclear region (ITS) to determine the genetic diversity of 199 accessions from 18 *Melilotus* species. The *rbc*L and *mat*K sequences were highly conserved, whereas the *trn*L-F and ITS sequences contained variable and parsimony-informative sites. In our analyses of the single and combined regions, we calculated the pairwise distance, haplotype and nucleotide diversity and gaps and then constructed phylogenetic trees to assess the genetic diversity, and our results revealed significant variations among the different accessions. The genetic distance values were between zero and nine, and based on the combined regions, the highest frequency value was approximately four. *Melilotus* showed high haplotype and nucleotide diversity, particularly in the ITS sequences, with values of 0.86 and 0.0087, respectively. The single ITS sequence, *psb*A-*trn*H, and the combined *mat*K+*rbc*L+*trn*L-F (MRT) and *mat*K+*rbc*L+*psb*A-*trn*H+*trn*L-F+ITS (MRPTI) regions showed interspecific variation in the gap analysis. Phylogenetic trees calculated using ITS, *psb*A-*trn*H and MRPTI sequences indicated distinct genetic relationship in 18 species, and these species could be divided into two groups. By determining the genetic diversity of plants, we can evaluate the genetic relationships among species and accessions, providing a basis for preserving and utilizing the genetic resources of *Melilotus*.

## Introduction

The genus *Melilotus* (sweet clover) consists of 19 annual and biennial species and belongs to the tribe Trifolieae of the legume family. Almost all species are native to North Africa or Eurasia, and manys can be found in North of China and Central Asia [1,2]. *Melilotus* is an important forage crop, and certain species, such as *M*. *albus*, *M*. *officinalis* and *M*. *indicus* have been cultivated in many regions [3]. Compared with other forages, the members of *Melilotus* can tolerate extreme environmental conditions, such as drought, cold, and high salinity [1,4], and its nitrogen fixation rate is higher than that of other legumes, which can increase soil fertility [5]. Additionally, *Melilotus* is valuable because of its coumarin content[6], and thus represents a possible medicinal plant resource. Due to its affordability and abundance as well as its potential market value, *Melilotus* is worthy of further investigation [6].

Genetic diversity within a particular species helps plants adapt to various environmental conditions, such as fluctuating climate and soil conditions; thus, assessing the diversity of available plant genetic resources is necessary to identify the genes associated with useful biological functions that can then be rationally integrated to design new varieties [7]. Plant genetic diversity has gained increasing attention because of the increase in human population as evidenced by rapid urbanization and the conversion of cultivable lands. These are the critical factors contributing to food insecurity in the developing world [8]. Consequently, the Consultative Group for International Agricultural Researches has begun establishing research centres and gene banks to conserve the plant genetic resources of staple food crops around the world, such as maize from Mexico, rice from North China and potatoes from Peru (for more information, see http://www.cigar.org/center/index.html).) The purpose of this organization is to maintain genetic diversity and to provide tools for population monitoring and assessment that can be used for conservation planning [9]. Forage crops also play an increasing role in farming system with the emphasis on development of sustainable agricultural production and the researches about genetic diversity on forage will assume greater importance for germplasm collections and breeding work [10,11]. Genetic diversity assessments are performed using morphological, biochemical and DNA marker analyses. Based on further studies on biological resources, improvements of molecular biology technology, the maturation of amplification and sequencing technologies, and decreases in costs, DNA markers have become the primary method of analysing genetic diversity. Currently, a wide range of DNA markers have been employed to assess genetic diversity, and these include random amplified polymorphic DNA (RAPD) has been adopted in bamboo [12], restriction fragment length polymorphisms (RFLPs) in rice [13], amplified fragment length polymorphisms (AFLPs) in walnuts [14], simple sequence repeats (SSRs) in potato [15], single nucleotide polymorphisms (SNPs) in wheat [16], and chloroplast DNA (cpDNA) in *Brassica napus* [17,18].

A previous study showed that the leaves, flower colour and structure, and pod and seed characteristics of *Melilotus* present extensive variation [19], and the agronomic and quality traits of 19 *Melilotus* species have been evaluated [20]. However, there is limited genetic information regarding *Melilotus* because previous research has concentrated on morphology, cultivation techniques and chemical composition, but SSR marker analyses have shown that *Melilotus* is highly diverse, which is indicative of high allelic richness in the accessions [21]. Understanding the genetic diversity of the plant will enable its genetic material to be preserved as a resources, such as in gene banks and DNA libraries [8]. Additionally, determining the genetic variability in crops provides useful information for breeders developing of new varieties. Cytoplasmic chloroplast genomes (cpDNA) have been widely employed as reference DNA to evaluate population-level genetic diversity [22]. Cytoplasmic chloroplast genomes isinherited highly conservatively in most angiosperms [23], and it has a simplex genome structure and shows vegetative segregation, intracellular selection, and reduced recombination [24,25]. The genetic diversities of *Brassica napus*, *Brassica rapa* and *Brassica oleracea* and their genetic relationships have been finely determined at the cpDNA level [17], and their cpDNA sequences have been used for determinations of genetic structure and population variability in genetic comparisons of Iranian Asafetida (*Ferula assa-foetida* L.) populations [26]. Accordingly, adopting several regions that cover nuclear DNA and cpDNA might be an effective strategy for evaluating genetic diversity [27,28]. To further study the genetic diversity of and acquire molecular data on *Melilotus*, we used five sequences, including *rbc*L, *mat*K, *psb*A-*trn*H and *trn*L-F and ITS, to assess the genetic diversity within 18 species.

## Materials and methods

### Plant materials

Seeds for sampling were selected from 151 accessions from the National Gene Bank of Forage Germplasm (NGBFG, China) and 48 accessions from the National Plant Germplasm System (NPGS, USA) for a total of 199 accessions representing 18 *Melilotus* species (S1 Table). The NGBFG accessions were mainly distributed in North China and adjacent areas such as Russia, whereas the NPGS accessions were mainly distributed in other regions. Because of their hardness, we rubbed the *Melilotus* seeds between two pieces of sand paper for 1 min, and the seeds were then germinated at 24°C after incubation over a 16-h light/8-h dark cycle. Ten days later, approximately 20 seedlings of each accession were collected and maintained at -80°C until assayed.

### DNA extraction, amplification, and sequencing

Total genomic DNA was extracted from whole seedlings using the SDS (sodium dodecyl sulphate) method [29]. For each accession, two to three DNA samples were extracted, and we selected one sample that revealed a proper DNA concentration for sequencing to minimize errors. Five sequences (four chloroplast regions, *rbc*L [30], *mat*K [31], *psb*A-*trn*H [32] and *trn*L-F [33] and one nuclear gene, ITS [34]) were amplified and sequenced (for the primer sequences, see S2 Table). Amplification was performed by polymerase chain reaction (PCR) in 25-μL mixtures containing 12.25 μL of 2×reaction mix, 0.25 μL of Golden DNA polymerase, 2 μL of each primer (1 μmol / mL), 2 μL of template genomic DNA (50 ng/mL) and 6.5 μL of deionized water as follows: 3 min at 94°C, 35 cycles of 30 s at 94°C, 30 s at 53°C, and 50 s at 72°C (the annealing temperature and extension time varied according to the sequences, see S2 Table), with a final extension of 7 min at 72°C before holding at 4°C. The amplified bands of the PCR products were validated by agarose gel electrophoresis and sequenced by Shanghai Shenggong Biotechnological, Ltd. (Shanghai, China).

### Data analyses

We used the Contig Express module of Vector NTI Suite 6.0 (InforMax, Inc) to assemble and edit the contigs [35]. Sequences were aligned using DNAMAN 7.0 [36], and the nucleotide variations were then determined. To calculate the average distances and gaps among the 18 species, several sequences were combined, and the combinations of each accession were assembled such that all sequences were connected end to end in the same order. The genetic diversity of *Melilotus* was analysed using DnaSP software, and we estimated the genetic diversity of the species based on the five sequences by calculating the pairwise distances for each locus using MEGA 6.0 according to the number of differences model [37]. In addition, the Emboss Needle algorithm (http://www.ebi.ac.uk/Tools/psa/emboss_needle/nucleotide.html) was employed to analyse the dissimilarities in nucleotide deletions via a pairwise sequence alignment [38]. We used Bayesian method to construct phylogenetic trees and *Vicia sativa* was adopted as outgroup [36].

## Results

DNA was extracted from 199 individuals representing 18 species of *Melilotus*. The results of the amplification were preliminarily validated by agarose gel electrophoresis (S1 Fig). We failed to obtain the PCR products of the *psb*A-*trn*H sequence in *M*. *italicus*. The PCR and sequencing success rates consistently exceeded 90% by optimizing the PCR amplification conditions.

### Alignment and DNA sequence data

The sequence length, GC content, variable sites and genetic distances based on the five sequences in 18 species were analysed and summarized (Tables 1–5, S3 Table). The lengths of the ITS, *mat*K, *rbc*L, *psb*A-*trn*H and *trn*L-F sequences were 691, 714, 756, 347 and 673 bp, respectively. Length variations occurred in each region, particularly in *trn*L-F, which ranged from 431 and 651 bp, but there was little length variation in the sequences of *mat*K and *rbc*L. Taken together, *M*. *albus*, *M*. *elegans*, *M*. *officinalis*, *M*. *polonicus* and *M*. *suaveolens* had similar sequence lengths. These species had different GC contents within the *psb*A-*trn*H and *trn*L-F sequences. The average GC content of *psb*A-*trn*H was 33.27%: *M*. *siculus* and *M*. *spicatus* had a higher than average GC contents, and *M*. *indicus* had the lowest GC content (31.66%). The average GC content of *trn*L-F was 33.28%. *Melilotus indicus* and *M*. *albus* had the highest and lowest GC contents, which were 34.60% and 31.56%, respectively.

**Table 1:** Sequence characteristics, pairwise distances and analyses of genome genetic diversity based on ITS sequences.

Species	Length (bp)	G+C Conten (%)	Intraspecific distance (mean)	Interspecific distance (mean)	Haplotype diversity (%)	Nucleotide diversity (%)
*M*. *ablus*	646	49.69	0.000	0~5.348 (1.860)	0.418±0.073	0.00076±0.00074
*M*. *altissimus*	650	49.33	0.000	1.862~5.522 (2.698)	0.833±0.222	0.00385±0.00199
*M*. *dentatus*	646	49.69	0.000	0~5.348 (1.860)	0.778±0.091	0.00169±0.00095
*M*. *elegans*	646	49.58	0~1.969 (1.217)	0~5.544 (2.188)	0.893±0.111	0.00348±0.00146
*M*. *hirsutus*	646	49.36	0~0.971 (0.647)	0~5.434 (1.921)	0.667±0.314	0.00206±0.00146
*M*. *indicus*	649	49.20	0~1.875 (1.234)	0~5.765 (3.558)	0.800±0.164	0.00339±0.00148
*M*. *infestus*	649/658	49.31	0.000	2.360~5.284 (4.446)	0.000	0.000
*M*. *italicus*	648	50.00	0.000	3.301~5.481 (3.694)	0.000	0.000
*M*. *officinalis*	646	49.48	0~1.371 (0.713)	0~5.479 (2.156)	0.710±0.079	0.00189±0.00093
*M*. *polonicus*	646	49.69	0.000	0~5.348 (1.860)	0.000	0.000
*M*. *segetails*	649/652	49.36	4.765	0~5.221 (3.694)	1.000±0.500	0.02946±0.0004567
*M*. *siculus*	654/655	49.84	0.986~3.120 (2.358)	2.303~5.765 (4.620)	1.000±0.500	0.00153±0.00153
*M*. *speciosus*	681	50.51	0.000	4.654~6.147 (4.679)	0.000	0.000
*M*. *spicatus*	647	49.40	0.000	2.505~5.316 (2.947)	0.500±0.265	0.00077±0.00084
*M*. *suaveolens*	646	49.63	0~1.641 (0.656)	0.942~5.594 (2.185)	0.529±0.117	0.00143±0.00110
*M*. *sulcatus*	655	49.46	0.000	2.303~5.266 (4.292)	0.000	0.000
*M*. *tauricus*	648	49.69	0.000	1.367~5.407 (2.355)	0.000	0.000
*M*. *wolgicus*	646	49.94	0~0.994 (0.397)	0.970~5.441 (2.231)	0.556±0.165	0.00129±0.00099
Average	691	49.62			0.861±0.024	0.00866±0.00255

ITS, internal transcribed spacer. The genetic diversity was analysed by a single sequence, and the same applies to the following tables.

**Table 2:** Sequence characteristics, pairwise distances and analyses of genome genetic diversity based on *mat*K sequences.

Species	Length (bp)	G+C Conten (%)	Intraspecific distance (mean)	Interspecific distance (mean)	Haplotype diversity (%)	Nucleotide diversity (%)
*M*. *ablus*	714	29.78	0~0.997 (0.598)	0~2.977 (1.525)	0.421±0.074	0.00074±0.00052
*M*. *altissimus*	714	29.69	0~1.380 (0.891)	0~2.779 (1.266)	0.833±0.222	0.00140±0.00108
*M*. *dentatus*	714	29.64	0.975~1.429 (1.133)	1.404~2.909 (2.008)	0.533±0.180	0.00177±0.00111
*M*. *elegans*	714	29.73	0~1.380 (0.733)	0~2.822 (1.247)	0.786±0.113	0.00170±0.0094
*M*. *hirsutus*	714	29.97	0.966~2.203 (1.716)	0~2.909 (1.989)	1.000±0.272	0.00467±0.00209
*M*. *indicus*	714	29.69	0~1.703 (1.076)	0~3.203 (1.510)	0.800±0.164	0.00224±0.00116
*M*. *infestus*	714	29.69	1.328~1.374 (1.348)	0~2.958 (1.461)	1.000±0.272	0.00280±0.00162
*M*. *italicus*	714	29.55	0.000	1.677~3.254 (2.048)	0.000	0.000
*M*. *officinalis*	714	29.64	0~1.437 (0.575)	0~2.872 (1.273)	0.518±0.122	0.00107±0.00076
*M*. *polonicus*	714	29.77	0~1.338 (0.535)	0~3.188 (1.282)	0.000	0.000
*M*. *segetails*	714	29.76	1.680	0~3.203 (1.501)	1.000±0.500	0.00420±0.00243
*M*. *siculus*	714	29.83	0~1.387 (0.925)	0.971~2.936 (2.388)	0.667±0.314	0.00187±0.00132
*M*. *speciosus*	714	29.76	1.420	2.737~3.623 (2.928)	1.000±0.500	0.00280±0.00198
*M*. *spicatus*	714	29.83	0.000	1.281~2.574 (1.910)	0.000	0.000
*M*. *suaveolens*	714	29.69	0~0.984 (0.394)	0~2.872 (1.230)	0.228±0.129	0.00033±0.00022
*M*. *sulcatus*	714	29.90	1.000	0.977~3.006 (2.280)	1.000±0.500	0.00140±0.00129
*M*. *tauricus*	714	29.69	0.000	0.958~2.539 (1.535)	0.000	0.000
*M*. *wolgicus*	714	29.83	0~1.934 (0.774)	1.010~2.962 (1.742)	0.222±0.166	0.00124±0.00103
Average	714	29.75			0.808±0.021	0.00294±0.00043

**Table 3:** Sequence characteristics, pairwise distances and analyses of genome genetic diversity based on *rbc*L sequences.

Species	Length (bp)	G+C Conten (%)	Intraspecific distance (mean)	Interspecific distance (mean)	Haplotype diversity (%)	Nucleotide diversity (%)
*M*. *ablus*	754	40.71	0.000	0~2.316 (0.659)	0.098±0.053	0.00013±0.00049
*M*. *altissimus*	754	40.71	0.000	0~2.316 (0.648)	0.000	0.000
*M*. *dentatus*	754	40.71	0.000	0~2.316 (0.638)	0.000	0.000
*M*. *elegans*	754	40.71	0.000	0~2.316 (0.659)	0.000	0.000
*M*. *hirsutus*	754	40.71	0.000	0~2.316 (0.638)	0.000	0.000
*M*. *indicus*	754	40.71	0.000	1.322~2.188 (1.571)	0.000	0.000
*M*. *infestus*	754	40.71	0.000	2.188~2.509 (2.319)	0.500±0.265	0.00332±0.00162
*M*. *italicus*	755	40.49	0.000	1.831~2.509 (1.936)	0.000	0.000
*M*. *officinalis*	755	40.71	0~0.978 (0.587)	0~2.316 (0.906)	0.228±0.102	0.00030±0.00036
*M*. *polonicus*	754	40.71	0.000	0~2.316 (0.659)	0.200±0.154	0.00027±0.00047
*M*. *segetails*	754	40.78	1.705	0~2.469 (1.477)	1.000±0.500	0.00398±0.00230
*M*. *siculus*	754	40.84	0.000	1.426~2.469 (1.533)	0.000	0.000
*M*. *speciosus*	754	40.58	0.000	1.293~2.212 (1.641)	0.000	0.000
*M*. *spicatus*	754	40.45	0.000	1.293~1.210 (1.624)	0.000	0.000
*M*. *suaveolens*	754	40.71	0.000	0~2.316 (0.659)	0.000	0.000
*M*. *sulcatus*	754	40.71	0.000	1.350~2.422 (1.486)	0.000	0.000
*M*. *tauricus*	754	40.71	0.000	0~2.316 (0.638)	0.000	0.000
*M*. *wolgicus*	754	40.71	0.000	0~2.316 (0.659)	0.000	0.000
Average	756	40.69			0.316±0.046	0.00117±0.00093

**Table 4:** Sequence characteristics, pairwise distances and analyses of genome genetic diversity based on *psb*A-*trn*H sequences.

Species	Length (bp)	G+C Conten (%)	Intraspecific distance (mean)	Interspecific distance (mean)	Haplotype diversity (%)	Nucleotide diversity (%)
*M*. *ablus*	318	33.64	0~1.410 (0.564)	0~3.238 (1.453)	0.163±0.065	0.00074±0.00066
*M*. *altissimus*	317/318	33.05	0~1.898 (1.229)	0~4.371 (1.655)	0.500±0.265	0.00472±0.00373
*M*. *dentatus*	318/321	32.91	0.966~4.371 (3.190)	0~5.278 (2.381)	0.222±0.166	0.00070±0.00116
*M*. *elegans*	318	33.64	0.000	0~4.371 (1.324)	0.250±0.180	0.00157±0.00172
*M*. *hirsutus*	318/319	32.88	0~0.966 (0.644)	0~4.371 (1.431)	0.667±0.314	0.00210±0.00210
*M*. *indicus*	319	31.66	0.000	1.660~4.590 (2.274)	0.000	0.000
*M*. *infestus*	317/318	33.68	0~1.412 (1.100)	0.929~4.786 (2.548)	0.883±0.222	0.00470±0.00275
*M*. *officinalis*	318	33.54	0~1.410 (0.564)	0~4.371 (1.450)	0.239±0.113	0.00155±0.00188
*M*. *polonicus*	318	33.64	0~1.344 (0.537)	0~4.371 (1.449)	0.378±0.181	0.00189±0.00193
*M*. *segetails*	318/319	32.65	0.000	0.988~4.333 (1.794)		
*M*. *siculus*	318	34.38	2.323~3.357 (2.610)	2.704~5.278 (3.323)	1.000±0.272	0.02516±0.01612
*M*. *speciosus*	304	32.89	0.000	0.929~4.577 (2.191)	0.000	0.000
*M*. *spicatus*	309/318	33.75	0~3.328 (2.159)	0~5.189 (2.342)	0.000	0.000
*M*. *suaveolens*	318	33.64	0~0.967 (0.387)	0~4.644 (1.624)	0.366±0.112	0.00115±0.00091
*M*. *sulcatus*	318	33.64	0.000	1.389~4.644 (2.338)	0.000	0.000
*M*. *tauricus*	318	33.33	0.000	0.982~4.518 (1.931)	0.000	0.000
*M*. *wolgicus*	322/334	32.72	0.000	0~4.347 (1.689)	0.000	0.000
Average	347	33.27			0.507±0.042	0.00643±0.00305

**Table 5:** Sequence characteristics, pairwise distances and analyses of genome genetic diversity based on *trn*L-F sequences.

Species	Length (bp)	G+C Conten (%)	Intraspecific distance (mean)	Interspecific distance (mean)	Haplotype diversity (%)	Nucleotide diversity (%)
*M*. *ablus*	432	31.56	0~4.143 (3.117)	0.965~8.074 (5.972)	0.667±0.163	0.02299±0.00409
*M*. *altissimus*	643	33.13	0~7.939 (3.969)	0~8.050 (4.755)	0.000	0.000
*M*. *dentatus*	639	33.02	0.000	0.940~8.060 (4.621)	0.000	0.000
*M*. *elegans*	431	32.10	1.300~4.282 (3.264)	0~8.076 (5.850)	1.000±0.177	0.02623±0.0579
*M*. *hirsutus*	657	33.49	0.000	1.887~8.107 (4.903)	0.000	0.000
*M*. *indicus*	442/612	34.60	0~7.112 (4.267)	0~8.129 (4.818)	0.000	0.000
*M*. *infestus*	442/646	33.13	0~7.106 (3.553)	0.981~8.095 (4.742)	0.000	0.000
*M*. *italicus*	617	34.36	0.000	2.393~8.102 (4.924)	0.000	0.000
*M*. *officinalis*	451	33.48	0~2.102 (1.402)	0~7.426 (5.289)	0.625±0.108	0.00420±0.00207
*M*. *polonicus*	452/453	33.26	0~2.121 (1.210)	0~7.459 (5.429)	0.524±0.209	0.00716±0.00255
*M*. *segetails*	612/655	33.97	2.195	1.876~8.092 (4.573)	1.000±0.500	0.0199±0.00574
*M*. *siculus*	653/654	33.21	0.000	0.943~8.147 (4.825)	0.000	0.000
*M*. *speciosus*	641	33.23	0.000	1.923~8.144 (4.841)	0.000	0.000
*M*. *spicatus*	452/607	34.39	0~7.428 (4.952)	0.935~8.099 (4.704)	0.000	0.000
*M*. *suaveolens*	432	32.60	0.968~4.266 (3.162)	0.935~8.144 (5.747)	1.000±0.052	0.02512±0.00429
*M*. *sulcatus*	647/656	32.85	2.291	2.062~8.122 (5.095)	1.000±0.500	0.00927±0.00379
*M*. *tauricus*	612/646	33.48	1.362~2.493 (1.995)	0~8.084 (4.723)	1.000±0.500	0.00310±0.0219
*M*. *wolgicus*	638	33.23	0.000	0~8.067 (4.467)	0.000	0.000
Average	673	33.28			0.965±0.009	0.12924±0.01834

The sequence diversity of the five loci in *Melilotus* was summarized, and the genetic diversity in each region of the 18 species was calculated (Tables 1–5, S2 Table). Analysis of the ITS sequences revealed 525 conserved sites and 121 variable sites, including 49 parsimony-informative sites and 72 single variable sites. *Melilotus elegans* and *M*. *altissimus* had high haplotype and nucleotide diversity. *Melilotus siculus* had high haplotype diversity but low nucleotide diversity. Analysis of the other four chloroplast regions showed that the haplotype and nucleotide diversities were lower than those of the ITS sequences. *Melilotus infestus* showed high diversity and *M*. *officinali*s had higher diversity than *M*. *albus*. Overall, *Melilotus* showed high haplotype and nucleotide variation in the ITS and *mat*K sequences. Several species, such as *M*. *tauricus*, had low diversity in most sequences.

### Genetic distance and similarity

To determine the average distances among the 18 species, we combined several sequences to calculate the pairwise distances (Fig 1). These combinations included *mat*K+*trn*L-F (MT), *mat*K+*rbc*L+*trn*L-F (MRT), *mat*K+*rbc*L+*psb*A-*trn*H+*trn*L-F (MRPT), *mat*K+*rbc*L+ITS+*trn*L-F (MRIT), and *mat*K+*rbc*L+*psb*A-*trn*H+*trn*L-F+ITS (MRPTI). Our results revealed that the highest frequency was approximately four in all combinations. The genetic distance value ranged from zero to nine according to the different accessions. For the five single regions, more than half of the species exhibited zero intraspecific distances within the ITS and *mat*K sequences. Several species, including *M*. *albus*, *M*. *italicus*, *M*. *officinalis*, *M*. *polonicus*, *M*. *speciosus* and *M*. *tauricus*, showed small intraspecific distances. *M*. *indicus*, *M*. *infestus*, *M*. *italicus*, *M*. *siculus*, *M*. *speciosus* and *M*. *sulcatus* had similar interspecific distances because of the large distances between these species calculated using four loci (except *trn*L-F, which presented high interspecific distances in all species).

**Fig 1:** Genetic distance histograms for five combined regions (*mat*K+*trn*L-H, MT; *mat*K+*rbc*L+*trn*L-H, MRT; *mat*K+*rbc*L+*psb*A-*trn*H+*trn*L-H, MRPT; *mat*K+*rbc*L+ITS+*trn*L-H, MRIT; *mat*K+*rbc*L+*psb*A-*trn*H+*trn*L-H+ITS, MRPTI). The dataset from this study was obtained with MEGA 6.0 Compute Pairwise Distance, and the histograms were generated using R 3.2.3.

Furthermore, we calculated the similarity, gaps and scores through a pairwise sequence alignment to analyse the intraspecific and interspecific divergence (Figs 2 and 3). We observed few nucleotide deletions in *mat*K and *rbc*L, zero gaps, and approximately 100% similarity. A diversity of gaps was observed in the other three single sequences and combined regions. The intraspecific gap value of *M*. *infestus* and *M*. *segetalis* was large in the ITS sequence and close to zero in the other sequences. Approximately half of the species showed differences in interspecific gaps. *M*. *speciosus* had the highest gap value of 0.069. According to the alignment of *psb*A-*trn*H, almost all species showed variations in interspecific gaps. The four species, *M*. *dentatus*, *M*. *segetalis*, *M*. *spicatus* and *M*. *wolgicus*, showed high intraspecific diversity in gap values. For the *trn*L-F sequence, the intraspecific gap value was higher in *M*. *altissimus*, *M*. *indicus*, *M*. *infestus* and *M*. *spicatus*, and all species showed high interspecific variation. Only a small difference in the interspecific gap value was observed among the 18 species based on the five sequences except in *M*. *dentatus*. After removing the *trn*L-F sequence, the variation was apparent. A higher diversity was found after removing the ITS and *psb*A-*trn*H sequences. To a certain extent, the gap value could reveal the diversity among the sequences in 18 species.

**Fig 2:** Average intraspecific gene gap value for single and combined regions based on the analysis of hundreds of sequences by pairwise sequence alignment. ITS, internal transcribed spacer.

**Fig 3:** Average interspecific gene gap value for single and combined regions based on the analysis of hundreds of sequences by pairwise sequence alignment.

### Cluster analysis

Based on genetic distance and similarity analysis, the ITS and *psb*A-*trn*H showed high discriminating in *Melilotus*. And phylogenetic trees were constructed using the Bayesian method based on the ITS, *psb*A-*trn*H respectively, and a combined region of the five sequences (Figs 4 and 5, S2 Fig). According to the Bayesian trees, all species showed distinct diversity with little mixing and we could divided 18 species into two groups on the basic of clades and branch length in Figs 4 and 5. The first group included *M*. *albus*, *M*. *altissimus*, *M*. *dentatus*, *M*. *elegans*, *M*. *hirsutus*, *M*. *officinalis*, *M*. *polonicus*, *M*. *segetalis*, *M*. *suaveolens*, *M*. *tauricus* and *M*. *wolgicus*. The second group contained the others. Similar to the analysis of genetic diversity, *M*. *albus*, *M*. *officinalis*, *M*. *tauricus* and *M*. *polonicus* showed small intraspecific distances since there are few clades among them. What’s more, the species in the first group have a closer genetic relationship due to similar branch length. The variation was smaller when we combined five sequences (S2 Fig). But we also could find the differences of accessions from different regions. Five accessions of *M*. *albus* from NPGS (USA) didn’t get together with other accessions from NGBFG (China). And accessions from the same area tend to be together, such as Mo_CF… and Mo_PI… in *M*. *officinalis*.

**Fig 4:** Bayesian tree with branch length, based on *psb*A-*trn*H sequences. The abbreviations represent 18 species: Ma—*M*. *albus*, Mm—*M*. *altissimus*, Md—*M*. *dentatus*, Me—*M*. *elegans*, Mh—*M*. *hirsutus*, Mi—*M*. *indicus*, Mf—*M*. *infestus*, Mr—*M*. *italicus*, Mo—*M*. *officinalis*, Mp—*M*. *polonicus*, Mg—*M*. *segetalis*, Mc—*M*. *siculus*, Ms—*M*. *speciosus*, Mu—*M*. *spicatus*, Mn—*M*. *suaveolens*, Ml—*M*. *sulcatus*, Mt—*M*. *tauricus*, and Mw—*M*. *wolgicus*. See S1 Table for the accession numbers.

**Fig 5:** Bayesian tree with branch length, based on ITS sequences. The abbreviations represent 18 species: Ma—*M*. *albus*, Mm—*M*. *altissimus*, Md—*M*. *dentatus*, Me—*M*. *elegans*, Mh—*M*. *hirsutus*, Mi—*M*. *indicus*, Mf—*M*. *infestus*, Mr—*M*. *italicus*, Mo—*M*. *officinalis*, Mp—*M*. *polonicus*, Mg—*M*. *segetalis*, Mc—*M*. *siculus*, Ms—*M*. *speciosus*, Mu—*M*. *spicatus*, Mn—*M*. *suaveolens*, Ml—*M*. *sulcatus*, Mt—*M*. *tauricus*, and Mw—*M*. *wolgicus*.

## Discussion

*Melilotus* is an important forage and green manure crop with high protein content and the ability to fix nitrogen [39], and it also plays an important role in soil improvement, is drought resistant and moderately winter hardy, and has good dry matter production [40,41]. However, there is limited information regarding its morphology, cultivation techniques and chemical composition; thus, genetic diversity analyses based on five sequences were performed in this study to provide a reference for the conservation of genetic resources.

As shown in Tables 1–5 and S2 Table, the *trn*L-F and ITS sequences provided more variation sites and informative characteristics than the other three sequences. Many studies have reported that ITS sequences have more variable and informative sites than cpDNA [32,42]: White (1990) found that the ITS sequence conserved its length and presented high nucleotide variability [43]. Chloroplast DNA, which is conservatively inherited, has a simple genome structure [17] and presents differences among populations and individuals in many species [44,45]. Due to differences in length, the *trn*L-F region contained more variation sites and greater genetic distances than the other regions in this study. The *rbc*L and *mat*K sequences were highly conserved in *Melilotus*, and the similarity among accessions was greater than 99.20% and 98.60%, respectively. The analysis of the five loci showed that the ITS and *psb*A-*trn*H sequences had more genetic diversity in *Melilotus*, whereas *rbc*L and *mat*K could be used in combination with other sequences. In addition, the intraspecific and interspecific distances calculated using the *rbc*L and *mat*K sequences were smaller than those of the other sequences. Our results were similar to the findings obtained by Chen, Yao et al [46], who found that the order of the sequences according to the interspecific distance value (from large to small) was ITS, *psb*A-*trn*H, *mat*K and *rbc*L. Previous researches showed that the *rbc*L and *mat*K sequences were suitable for analyzing relationship at higher taxonomic levels [47,48], and when assessing genetic diversity at the species or genus level, the ITS and *psb*A-*trn*H sequences worked better and the combination of several sequences vielded the best result. Moreover, the sequence characteristics in *Melilotus* could be used in further genetic diversity studies.

Our previous study showed that the SSR marker analysis revealed highly significant differences in genetic differentiation among accessions within *Melilotus* species accessions [21]. According to the haplotype and nucleotide diversity calculated using the five sequences, *Melilotus* showed higher diversity, particularly within the ITS sequences, than *Euphrasia* and *Rhododendron* [49,50], which had a haplotype and nucleotide diversity of 0.86 and 0.0087, respectively. The analysis of gaps in the 18 species revealed a high degree of variation based on the ITS, *psb*A-*trn*H and combined MRT and MRPI sequences. Additionally, the distance in *Melilotus* was significantly higher than that in species of *Rhodiola* [32] calculated using ITS, *rbc*L, *mat*K and *psb*A-*trn*H regions. Compared with *Medicago sativa*, *Melilotus* has not been cultivated commercially and shows higher diversity [21,51]. In addition, cluster analysis divided 18 species into two groups, which is similar to the results of previous studies [21,34]. Traditional identification depends on the shape of the torus and flower colour [52], but plant morphology might vary greatly within a single plant [53]. This research divided *Melilotus* into two groups according to flower colour. The white group contains four species, *M*. *albus*, *M*. *tauricus*, *M*. *wolgicus* and *M*. *speciosus*, and the other species composed the yellow group [53]. However, due to differences in the result of these molecular studies, flower colour has no obvious link with the phylogenetic classification [34] and might not be a reliable basic for classification. Compared with the results in previous studies [21,34], *M*. *albus*, *M*. *altissimus*, *M*. *elegans*, *M*. *officinalis*, *M*. *polonicus*, *M*. *suaveolens*, *M*. *wolgicus* were included in the first group and *M*. *italicus*, *M*. *speciosus*, *M*. *siculus*, *M*. *indicus*, *M*. *sulcatus*, *M*. *infestus*, *M*. *spicatus* were included in the second group. These *Melilotus* species clustering within the same group may have closer genetic relationships.

The significant differences were revealed among *Melilotus* species, and several, such as *M*. *infestus* and *M*. *segetails*, showed higher diversity than the others. To reduce the loss of *Melilotus* genetic resources, it is necessary to strengthen the collection and protection of wild germplasm resources. Current situation of the conservation of genetic resources in *Melilotus* is too many individuals of *M*. *albus* and *M*. *officinalis* were collected but the germplasm collections of other species were insufficient. Imbalance of these species is the main problem we are facing in germplasm collection and conservation. Surveys should occur worldwide and more individuals of the species with high diversity revealed by Tables 1–5 might need to be collected. The growing population pressure and urbanization of agricultural lands as well as the rapid modernization of every aspect of our day-to-day activities have caused biodiversity decreased in directly and indirectly, and the large-scale cultivation of genetically homogenous varieties also reduces species diversity and genetic variation [54]. What’s more, this study identified additional *Melilotus* genetic resources for breeding purpose. The loss of genetic diversity has been recognized as the result of a genetic bottleneck imposed on crop plants during domestication and by modern plant-breeding practices [55]; thus, this research could provide a reference for the conservation of genetic resources that currently exist for the future breeding work.

Our results identified the characteristics of five sequences in *Melilotus* and indicated that analyses of these regions represent a valuable method for assessing genetic diversity. The analysis of the five loci provided important genetic information that will assist in germplasm collection and conservation of *Melilotus*.

## Supporting information

S1 Fig Electrophoretogram of the PCR amplifications based on five sequences. From one to eighteen: *M*. *albus*, *M*. *altissimus*, *M*. *dentatus*, *M*. *elegans*, *M*. *hirsutus*, *M*. *indicus*, *M*. *infestus*, *M*. *italicus*, *M*. *officinalis*, *M*. *polonicus*, *M*. *segetalis*, *M*. *siculus*, *M*. *speciosus*, *M*. *spicatus*, *M*. *suaveolens*, *M*. *sulcatus*, *M*. *tauricus*, and *M*. *wolgicus*.
(TIF)

S2 Fig Bayesian tree based on the combined regions of five sequences. The abbreviations represent 18 species: Ma-*M*. *albus*, Mm-*M*. *altissimus*, Md-*M*. *dentatus*, Me-*M*. *elegans*, Mh-*M*. *hirsutus*, Mi-*M*. *indicus*, Mf-*M*. *infestus*, Mr-*M*. *italicus*, Mo-*M*. *officinalis*, Mp-*M*. *polonicus*, Mg-*M*. *segetalis*, Mc-*M*. *siculus*, Ms-*M*. *speciosus*, Mu-*M*. *spicatus*, Mn-*M*. *suaveolens*, Ml-*M*. *sulcatus*, Mt-*M*. *tauricus*, Mw-*M*. *wolgicus*. See S1 Table for the accession number.
(TIF)

S1 Table Information on the 199 *Melilotus* accessions included in this study. (XLS)

S2 Table Information on the primers, amplification conditions and sequence statistics for the five sequences. (XLS)

S3 Table Variable sites of the five sequences in the 18 species. The four colours represent the four canonical bases: green for adenine (A), blue for cytosine (C), purple for guanine (G) and orange-red for thymine (T). The symbol “▲” represents the sequence deletions from 1 to 188.
(XLS)
